# Neuroendocrine neoplasm with metastasis to the thyroid: a case report and literature review

**DOI:** 10.3389/fonc.2023.1024908

**Published:** 2023-04-28

**Authors:** Yu Zhang, Bei Lin, Kai-ning Lu, Yue-ping Teng, Tian-han Zhou, Jia-yang Da, Fan Wu, Gang Pan, Ding-cun Luo

**Affiliations:** ^1^ Department of Oncological Surgery, Affiliated Hangzhou First People’s Hospital, Zhejiang University School of Medicine, Hangzhou, Zhejiang, China; ^2^ The Fourth School of Clinical Medicine, Zhejiang Chinese Medical University, Hangzhou, Zhejiang, China; ^3^ Department of Breast Surgery, First Affiliated Hospital of Nanjing Medical University, Nanjing, China; ^4^ Department of Operating Room, Affiliated Hangzhou First People’s Hospital, Zhejiang University School of Medicine, Hangzhou, Zhejiang, China; ^5^ Department of General Surgery, Zhejiang Provincial Hospital of Chinese Medicine, Hangzhou, Zhejiang, China; ^6^ Department of Dermatology, Third People's Hospital of Hangzhou, Hangzhou, China

**Keywords:** neuroendocrine tumor, neoplasm metastasis, thyroid gland, rectal cancer, FNA

## Abstract

Thyroid cancer can be divided into two types according to its cellular origin, i.e., malignant tumors originating from thyroid cells and cancers that metastasize to the thyroid from other sites, the latter of which are, clinically rare. This article reports the diagnosis and treatment of a rectal neuroendocrine neoplasm metastasis to the thyroid. No similar cases have been reported before. This case suggests that when evaluating thyroid tumors, clinicians should not only carefully identify the clinical features of the tumor but also pay special attention to the patient’s history of tumors, especially neuroendocrine neoplasms. For definite secondary thyroid malignancies, neck surgery is feasible if the thyroid is the only site of metastasis; otherwise, the subsequent diagnosis and treatment plan should be determined after a comprehensive evaluation of the primary tumor and patient’s general condition.

## 1 Introduction

Thyroid metastases (TMs) refer to a class of diseases that metastasize from nonthyroid malignancies to the thyroid. A retrospective study by Ghossein CA (1) found that the incidence of TM was 0.36% among all patients with thyroid malignancies who visited the center from 2003 to 2019. According to Tang Q (2), who reviewed the literature from 1979 to 2021, the most common origins of metastasis in these patients were renal cell carcinoma (48.1%), colorectal cancer (10.4%), lung cancer (8.3%), breast cancer (7.8%) and sarcoma (4.0%). The majority of colorectal cancer metastases to the thyroid originate from colorectal adenocarcinoma (3–5), and no cases of metastasis from rectal neuroendocrine neoplasms (NENs) to the thyroid gland have been reported. Herein, we report a case of rectal NEN metastasis to the thyroid and discuss the diagnosis and treatment of this patient. This study aims to improve clinicians’ ability to diagnose and treat TM and improve patient survival rate and quality of life.

## 2 Case report

A 56-year-old woman presented with neck pain 1 month after the discovery of a thyroid nodule that developed 1 year prior. The patient was first found to have thyroid nodules by ultrasound in August 2017 (the details are unknown), and there were no symptoms of compression, hoarseness, palpitation, low-grade fever, or choking at that time. However, as the patient was only three months post-rectal cancer surgery and had a significant reaction to chemotherapy, she was extremely weak. The patient and their family chose to have regular follow-up examinations without further treatment for the thyroid nodules. Through regular follow-ups, the thyroid nodules grew larger and were accompanied by mild neck pain and enlarged surrounding lymph nodes. Therefore, the patient came to our hospital for further examination In September 2018, the patient came to the clinic after experiencing neck pain without other obvious discomfort. When palpating the thyroid gland in this patient, bilateral hard masses could be felt, measuring approximately 1.5*1.5 cm in size, with an unclear boundary, tenderness and rigidity, and the masses moved up and down with swallowing. Moreover, swollen and hard lymph nodes could be palpated on both sides of the neck, with a maximum size of approximately 2.0*1.0 cm. The rest of the physical examination showed no obvious abnormalities. Color Doppler ultrasound (**Figure 1**) and computed tomography (CT) showed multiple nodules with increased signals in the bilateral lobes of the patient’s thyroid; among them, the largest nodule on the right side was 2.0*2.0 cm and the largest nodule on the left side was 1.0*1.5 cm. The results of routine laboratory tests, including for those for thyroid function (T3, T4, TSH), liver and kidney function, and tumor markers (AFP, CEA, CA-199, CA-125, CA-153, CA-242), were normal. To further clarify the condition of the patient’s lesions, we performed a puncture biopsy. Fine-needle aspiration (FNA) revealed the presence of suspicious tumor cells in the left thyroid nodule and infiltration or metastasis of malignant tumor cells in the left cervical lymph nodes. In May 2017, the patient underwent enteroscopy because bloody stools for 8 months and aggravated for the last 2 months. The result of enteroscopy suggested a rectal mass (**Figure 2A**) and the patient had previously undergone radical rectal resection for a rectal neuroendocrine neoplasm (NEN). The postoperative pathology showed a neuroendocrine tumor (**Figure 2B**), with a tumor size of 3.1cm*2.5cm, and the immunohistochemical results showed CK7[-], CK20[focal +], CKpan[+], Syn[+], CgA[-], CDX2[-], CD56[+], Ki67[5-10%], and EMA[partially+]. The postoperative pathology showed that the endocrine tumor of the rectum was a well-differentiated neuroendocrine tumor, WHO grade 2 (G2), stage IIIB. Chemotherapy with etoposide 120 mg + cisplatin 60 mg (EP regimen) was given for two cycles one month after surgery. The patient failed to continue chemotherapy due to personal reasons, and no abnormalities were found in subsequent reexaminations. Since the patient had no other distant metastatic lesions, we performed bilateral total thyroidectomy + bilateral central lymph node dissection on October 31, 2018. Postoperative pathology suggested bilateral metastatic thyroid NENs (**Figure 3**) and the immunohistochemical results showed CK[+], TG[-], TTF1 slightly scattered[+], HBME-1[-], S-100[-], Calcitonin[-], CgA[+], Syn[+], Ki-67[+] 10-20%, CK19 [+], CK20[-], PAX 8[-], CEA[-], CDX2[-] and SATB2[-] (**Figure 4**).

**Figure 1:** Ultrasound image and blood flow diagram of the patient’s lesion. **(A)** Ultrasound showed that there was an isoechoic nodule in the right lobe of the patient, with a size of approximately 2*2 cm, a regular shape, and an uneven halo around the edge. **(B)** Blood flow map showed poor blood flow in the patient’s right nodule. **(C)** Ultrasound showed that there was an isoechoic nodule in the right lobe of the patient, approximately 1.5*1 cm in size, with a regular shape and an uneven halo around the edge. **(D)** The blood flow map showed that the patient’s left nodule did not have rich blood flow.

**Figure 2:** The patient’s preoperative colonoscopy images and pathological images of rectal tumors. **(A)** The patient’s preoperative colonoscopy images. **(B)** The patient’s preoperative pathological images of rectal tumors.

**Figure 3:** Histological findings of a rectal neuroendocrine tumor metastasized to the thyroid. **(A)** Rectal neuroendocrine tumors are indicated by white arrows, and normal thyroid epithelial cells are indicated by black arrows (HE; 100X). **(B)** Metastatic neuroendocrine tumor without normal thyroid tissue (HE; 400X).

**Figure 4:** Immunohistochemical and cytological evidence of rectal neuroendocrine tumor metastasis to the thyroid. **(A)** Cancer cells negative for S-100 (S-100; 400X). **(B)** HE staining demonstrated typical neuroendocrine tumor morphology (HE; 400X). **(C)** Cancer cells positive for CgA (CgA; 400X). **(D)** Cancer cells positive for Syn (Syn; 400X).

The patient underwent regular follow-up after surgery. In January 2019, liver metastases were detected in another examination, followed by multiple metastases in bone and the pelvis. Oxaliplatin 130 mg D1+ S-1 60 mg d1-7 (SOX), anlotinib, irinotecan 260 mg d1 q2w and other drugs were used successively. Ultimately, the patient died of liver metastasis in May 2022, but there was no sign of recurrence in the neck.

## 3 Discussion

### 3.1 Epidemiology of metastatic thyroid carcinoma

Although the thyroid has an abundant blood supply, metastatic thyroid cancer is extremely rare (1, 6, 7). R.A. Willis (8) proposed two hypotheses to explain this phenomenon: 1. The faster blood flow in the thyroid prevents the adhesion of cancer cells. 2. The high oxygen saturation and high iodine content of the thyroid gland are not conducive to the growth of cancer cells. Metastatic cancer often occurs in thyroid tissue with existing lesions, such as Hashimoto’s thyroiditis, nodular goiter, and follicular adenoma. These basic lesions lead to changes in the thyroid microenvironment, which may create favorable conditions for the growth of metastatic cancer cells. However, there was no basic thyroid disease in this patient, so the cause of metastasis in this patient needs to be further explored. Moreover, the TMs in this patient were from a rectal neuroendocrine tumor, which is different from previous reports; thus, this case report has certain significance as a reference (9).

### 3.2 Epidemiology of rectal neuroendocrine tumors

NENs are rare and highly heterogeneous tumors originating from neuroendocrine organs or cells. The most common site of occurrence is the gastrointestinal tract, and rectal NENs are more common in Asian people. The latest domestic research data in Japan show that rectal NENs account for 53% (10) of all gastrointestinal tract NENs, which is much higher than the rate of 28.6% in the United States (11). The data of 11,329 patients with NENs in the US SEER database between 1988 and 2012 showed a distant metastasis rate of 2% for tumors with a diameter ≤10 mm, 2.4% for those with a diameter 11-19 mm, and 12% for those with a diameter ≥20 mm. Therefore, clinicians, especially those in Asia, should pay attention to the existence of rectal NENs and the risk of distant metastasis.

### 3.3 Diagnosis of metastatic thyroid carcinoma

TM has an insidious onset and often has no obvious clinical symptoms. Some patients may develop such tumors decades after the primary tumor is resected (12). Therefore, clinicians should remain alert to the possibility of metastatic thyroid cancer in patients with a history of malignancy and thyroid nodules. Color Doppler ultrasonography is the primary method recommended by domestic and foreign guidelines for the diagnosis of thyroid nodules, and this modality can also play an important role in the diagnosis of TMs. TMs have similar ultrasound characteristics similar to those of primary lesions, but their manifestations are diverse; they most commonly present as thyroid nodules or even areas with diffuse and uneven echogenicity. The main ultrasonographic manifestations of nodules are as follows: multiple lesions, large size, unclear boundary, irregular shape, solid, hypoechoic, calcification, and rich blood flow (13). In contrast to the above conclusions, the ultrasound images of this patient showed isoechoic nodules with clear boundaries, a regular shape, an uneven solid halo around the edge, and poor blood flow, which may be related to the different characteristics of the primary tumor. There was a high risk of misdiagnosis based on the B-mode ultrasound image of this patient, and such metastases should be carefully differentiated from the primary thyroid tumor and comprehensively judged based on the patient’s medical history. Fine-needle aspiration cytology (FNAC) is the first choice for patients with suspected metastatic thyroid cancer. FNAC is simple and easy to perform, and it is the best method for preoperative diagnosis (9). A multi-institution study report on FNAC showed that 87% of TM patients could be diagnosed with thyroid malignancy by FNAC, and 93% of them could be specifically diagnosed with TM (14). In this paper, preoperative FNAC indicated the possibility of malignancy, which provided an important basis for clinical decision-making. In conclusion, the diagnosis of TM should be based on ultrasound, FNAC and the patient’s past medical history.

### 3.4 Treatment

Due to the very low incidence of TM, there are still no guidelines for its treatment. Most scholars believe that to achieve local neck control or even a cure, surgical treatment is the priority for patients whose thyroid is the only site of metastasis and whose primary cancer can be resected and cured (15–17). Considering that there was no evidence of distant metastasis, bilateral thyroid nodules were present, and the possibility of malignancy was confirmed by left puncture, bilateral total thyroidectomy and bilateral central lymph node dissection were performed for this patient at our hospital. Although the patient had multiple systemic metastases after surgery, there was no obvious recurrence in the neck, and a local cure was achieved, which was consistent with the above literature. It is worth noting that most TM patients have multiple systemic metastases at the same time (18–20), and a study by Stergianos S (21) noted out that 81% of patients will have metastases in parts of the body other than the thyroid. The author believes that when TM occurs, it likely indicates that the human body is under a high tumor burden, and that probability of multiple metastases throughout the body is high. Therefore, it is recommended that regular and timely general examinations be conducted after the discovery of TM and that the frequency of examinations should be increased. If the patient has multiple systemic metastases, treatment should be considered according to the primary lesion and the site of metastasis.

### 3.5 Prognosis

The prognosis of TM remains controversial. Most scholars believe that the prognosis of TM is generally poor. The median survival time reported in previous literature is 8.8-34.0 months (15, 21, 22), and the five-year overall survival rate is 11%-58% (1, 23, 24). Factors associated with prognosis include the type of primary tumor (20) and the occurrence time, number, size, and location of the metastatic tumors (25). For example, Stergianos S (21) reported that the survival rate of TM patients was higher when the primary tumor was renal cell carcinoma, versus other types of primary tumors. This may be related to renal cell carcinoma having a low degree of invasiveness and malignancy. A report by Beutner U (26) also posted that the median survival time of TM patients with renal cell carcinoma was 6.5 years after active surgical treatment, while the median survival time of TM patients with other primary tumors was only 4.7 years after surgical treatment. However, Papi G (27) believed that the overall survival time of cancer patients was not correlated with the presence or absence of TM. In summary, the prognosis of TM needs to be confirmed with more long-term follow-up data from large-scale, multicenter studies.

In conclusion, clinicians should remain alert to the possibility of TM in patients with thyroid nodules and a history of other malignancies to avoid missed diagnosis, misdiagnosis, and delayed treatment. Additionally, B-mode ultrasound and FNAC are important methods to assist clinicians in the diagnosis of TM. Furthermore, clinicians should consider the risk of multiple systemic metastases when patients present with TM, and surgical treatment is a good option for patients with only TM. However, for patients with multiple metastases, the choice of local surgery or comprehensive systemic treatment needs to be further verified by more follow-up data from large-sample, multicenter studies.

## Data availability statement

The original contributions presented in the study are included in the article/supplementary material. Further inquiries can be directed to the corresponding author.

## Ethics statement

Informed consent was obtained from the participant/patient(s) for the publication of this case report.

## Author contributions

YZ: Conceptualization, Methodology, Resources, Formal analysis, Writing - Review & Editing. BL: Writing - Review & Editing. K-NL: Conceptualization, Methodology, Formal analysis, Resources, Writing - Original Draft. Y-PT: Resources, Data Curation, Writing - Review & Editing, Supervision. T-HZ: Resources, Data Curation, Supervision. J-YD: Formal analysis, Resources, Data Curation. FW: Formal analysis, Resources. GP: Resources, Data Curation, Writing - Review & Editing. D-CL: Resources, Supervision, Project administration, Writing - Review & Editing, Funding acquisition. All authors contributed to the article and approved the submitted version.
